# Daily Physical Activity Assessed by a Triaxial Accelerometer Is Beneficially Associated with Waist Circumference, Serum Triglycerides, and Insulin Resistance in Japanese Patients with Prediabetes or Untreated Early Type 2 Diabetes

**DOI:** 10.1155/2015/526201

**Published:** 2015-05-10

**Authors:** Hidetaka Hamasaki, Mitsuhiko Noda, Sumie Moriyama, Reo Yoshikawa, Hisayuki Katsuyama, Akahito Sako, Shuichi Mishima, Masafumi Kakei, Osamu Ezaki, Hidekatsu Yanai

**Affiliations:** ^1^Department of Internal Medicine, National Center for Global Health and Medicine Kohnodai Hospital, Chiba 272-8516, Japan; ^2^General Internal Medicine, Community Healthcare Studies, Jichi Medical University Graduate School, Tochigi 329-0498, Japan; ^3^Department of Diabetes Research, Diabetes Research Center, National Center for Global Health and Medicine, Tokyo 162-8655, Japan; ^4^Department of Human Health and Design, Faculty of Human Life and Environmental Sciences, Showa Women's University, Tokyo 154-8533, Japan

## Abstract

*Aim*. To investigate the association between daily physical activity and metabolic risk factors in Japanese adults with prediabetes or untreated early type 2 diabetes (T2D). *Methods*. Daily physical activity level was measured using a triaxial accelerometer. We assessed correlations between physical activity level and waist circumference, blood pressure, fasting levels of plasma glucose, serum triglycerides, and insulin and homeostasis model assessment-insulin resistance (HOMA-IR). *Results*. A total of 80 patients were studied. After adjustment for age and body mass index, in all subjects, physical activity level was negatively associated with waist circumference (*β* = −0.124, *P* = 0.018) and fasting serum triglycerides (*β* = −0.239, *P* = 0.035), insulin (*β* = −0.224, *P* = 0.022). In men, physical activity level was negatively associated with systolic blood pressure (*β* = −0.351, *P* = 0.044), fasting plasma glucose (*β* = −0.369, *P* = 0.025) and insulin (*β* = −0.362, *P* = 0.012), and HOMA-IR (*β* = −0.371, *P* = 0.011). No significant associations were found between physical activity level and metabolic risk factors in women. *Conclusion*. Objectively measured daily physical activity is beneficially associated with waist circumference, serum triglycerides, and insulin resistance in individuals with prediabetes or untreated early T2D. (This trial is registered with UMIN000015774.)

## 1. Introduction

Decreased time spent in moderate-to-vigorous physical activity has been reported to be independently associated with the risk of metabolic syndrome and its metabolic components [1–6]. However, the studies reporting this finding were all limited by the self-reported nature of the physical activity levels (PALs) they measured. Accurate evaluation of physical activity is essential to investigate the associations between PAL and the various metabolic risk factors. Recently, a number of small and lightweight accelerometers have been developed and become available for objectively evaluating the amount and intensity of physical activity. In a study of Australian adults without known diabetes, time spent in light physical activity and sedentary activity, measured using a uniaxial accelerometer, was found to be significantly associated with waist circumference and clustered metabolic risks [7]. In another study of Australian adults without diagnosed diabetes, light physical activity measured using uniaxial accelerometer was shown to be favorably associated with 2 h plasma glucose, while sedentary time was unfavorably associated with it [8]. Furthermore, in a study of 258 adults with a family history of T2D, total body movement measured by uniaxial accelerometer was significantly and independently associated with fasting triglycerides, insulin, HDL, and clustered metabolic risks after adjustment for age, sex, and obesity [9]. Triaxial accelerometers have been developed, and clinical studies have demonstrated higher correlation coefficients between counts obtained with these triaxial accelerometers and the energy expenditure measured in a chamber than with the counts obtained with uniaxial accelerometers [10–13].

It is known that the main determinant of variability in total daily energy expenditure is light physical activity, such as washing dishes, cleaning the floor, and typing on a personal computer [14, 15]. The energy expenditure due to such physical activities, which is known as nonexercise activity thermogenesis (NEAT) and is defined as the energy expenditure due to daily physical activities other than volitional sports-like exercise or resistance training [16], has been reported to be associated with the risk of obesity [17]. However, the extent to which light physical activity, including NEAT, is associated with metabolic risk factors is unclear, especially in relation to patients with prediabetes or untreated early type 2 diabetes (T2D). We previously demonstrated that NEAT is favorably associated with insulin sensitivity, waist circumference, high-density lipoprotein (HDL) cholesterol, and blood pressure in patients with T2D [18], but our study was also limited by the analysis of subjective data; briefly the NEAT score was calculated from self-reported questionnaire score and thus may not have accurately represented true NEAT values. Accordingly, we decided to use a triaxial device to obtain objective measurements of daily physical activity such as NEAT in this study.

The aim of present study was to examine more objectively and precisely the associations between daily physical activity and various metabolic risk factors in impaired glucose metabolism; in this study, we used objectively measured triaxial accelerometer data to evaluate daily physical activity such as NEAT of Japanese adults with prediabetes or untreated early T2D.

## 2. Methods

### 2.1. Participants

The study protocol was approved by the Medical Ethics Committee of the National Center for Global Health and Medicine (Reference Number NCGM-G-001212), and all participants provided written informed consent to participate. This study was performed in accordance with the Declaration of Helsinki.

Between August 2012 and December 2013, we recruited outpatients with impaired glucose metabolism who did not take any hypoglycemic agents or cholesterol-lowering agents for this cross-sectional observational study. Individuals who engaged in sports-like exercise or resistance training were excluded to evaluate only daily physical activity except for such active physical activities. Patients with physical disability such as osteoarthritis, cardiovascular, and/or respiratory diseases were also excluded because such daily life difficulties affect the measurement of daily physical activity. At the first medical examination, we asked all participants not to take exercise except for daily physical activities which was confirmed after the study period. All subjects were instructed to consume a calorie-restricted diet of 25 to 30 kcal/kg per day as diet therapy for diabetes by certified nutritional educators and to continue the diet during study period.

T2D was diagnosed according to any of the following diagnostic criteria: serum levels of hemoglobin A1c (HbA1c) ≥6.5%, fasting plasma glucose (FPG) ≥126 mg/dL, casual plasma glucose ≥200 mg/dL, and 2 h plasma glucose after the 75 g oral glucose tolerance test (OGTT) ≥200 mg/dL [19]. Prediabetes including impaired fasting glucose (IFG) and impaired glucose tolerance (IGT) was diagnosed as follows: for IFG, FPG levels of 110 mg/dL to 125 mg/dL and 2 h plasma glucose levels after OGTT <140 mg/dL; for IGT, FPG levels <110 mg/dL and 2 h plasma glucose levels after OGTT of 140 mg/dL to 199 mg/dL [19].

### 2.2. Anthropometric and Physiological Measurements

Height and weight were measured using a rigid stadiometer and calibrated scales (DP-7100PW; Yamato Co., Ltd., Hyogo, Japan). Waist circumference around the navel was measured with a nylon anthropometric tape (Rotary Measure; Futaba Co., Ltd., Saitama, Japan). Body mass index (BMI) was calculated by dividing body weight in kilograms by the square of body height in meters. Blood pressure was measured using an automatic sphygmomanometer (HEM-762; Omron Co., Ltd., Kyoto, Japan).

### 2.3. Blood Samples

After a 12 h overnight fast, blood samples were taken from the antecubital vein and collected into tubes. FPG was measured by an enzymatic method (Glucose Assay Kit; Wako Pure Chemical Industries, Osaka, Japan). Serum insulin and HbA1c were measured by automated enzyme-linked immunosorbent assays (*E*-test TOSOH II; TOSOH, Tokyo, Japan) and high-performance liquid chromatography (HA-8180; Arkray, Tokyo, Japan), respectively. Total cholesterol, triglycerides, HDL cholesterol, and low-density lipoprotein (LDL) cholesterol were measured enzymatically using the following commercially available kits: Tcho-l, TG-LH (both from Wako Pure Chemical Industries), Cholestest N HDL, and Cholestest LDL (both from Daiichi Pure Chemicals, Tokyo, Japan), respectively. We calculated homeostasis model of assessment-insulin resistance (HOMA-IR) as the marker for insulin resistance by using FPG and insulin concentrations and the following equation: HOMA-IR = FPG (mg/dL) × fasting serum insulin (*μ*U/mL)/405 [20].

### 2.4. Physical Activity Level Measurements

Daily physical activity was measured using a triaxial accelerometer (Active Style Pro HJA-350IT; Omron Co., Ltd.; 74 × 46 × 34 mm, 60 g including batteries). Subjects wore the accelerometer at the left waist to record PALs. Anteroposterior, mediolateral, and vertical acceleration measurements were obtained during each physical activity at a frequency of 32 Hz at 12-bit resolution. Each of the three signals from the triaxial accelerometer was passed through a high-pass filter with a cut-off frequency of 0.7 Hz to remove the gravitational acceleration component. The ratios of unfiltered to filtered total acceleration and filtered vertical and horizontal acceleration were calculated to determine the cut-off value for the classification of locomotive activities and nonlocomotive activities such as household and occupational activities, which resulted in almost 100% accurate demarcation of 11 daily activities [10]. Metabolic equivalent values (METs) determined using the same triaxial accelerometer have been reported to be closely correlated with METs calculated using energy expenditure measured by indirect calorimetry [10, 21].

Subjects wore the accelerometer at the left waist for 7 consecutive days and were requested to wear the device at all times except during sleeping, bathing, and swimming. Activity data were stored on a minute-by-minute basis and downloaded to a personal computer for analysis. We excluded days in which subjects did not wear the accelerometer for more than 8 h from the data analysis.

Basal metabolic rate (BMR) was estimated using the following multiple regression equation including age, sex, height, and ideal body weight (IBW) as variables: BMR (kcal/day) = [(0.1283 + 0.0481 × IBW (kg) + 0.0234 × height (cm) − 0.0138 × age (years) − 0.5473 × sex coefficient (man: 1; woman: 2)) × 293] [22]. Total energy expenditure (TEE) was calculated using a regression equation with the METs determined using the triaxial accelerometer [21]. PAL was calculated as follows: PAL = TEE/BMR [23]. We calculated average values of PAL for at least 5 days on which the subjects wore the accelerometer for more than 8 h.

### 2.5. Statistical Analysis

Statistical analysis was performed using SPSS version 19 (IBM Co., Ltd., Chicago, IL). All values are expressed as the mean ± SD. Differences in physical and biochemical data between men and women were analyzed using the Mann-Whitney* U* test. Multiple regression analysis was performed to test the independent correlations between PAL and physical and biochemical data. Models were adjusted for the potential confounders of age and BMI. We divided subjects into men and women to investigate sex differences in the correlations between PAL and the metabolic risk factors. *P* values less than 0.05 were considered statistically significant.

## 3. Results

Table 1 shows the physical and biochemical characteristics of the 80 subjects enrolled (38 men and 42 women; mean age ± SD, 57.6 ± 13.6 years; age range: 27–80 years). Fifty-four subjects were classified as having early T2D that had not ever been treated, 17 and 19 of whom were classified as having IFG and IGT, respectively. Eighteen subjects (9 men, 9 women) had taken antihypertensive agents.

Height, weight, and BMR values were significantly higher in men than in women. Total cholesterol was significantly higher in women than in men. No significant sex differences were noted for age, BMI, waist circumference, systolic blood pressure, diastolic blood pressure, FPG, HbA1c, triglycerides, HDL cholesterol, LDL cholesterol, serum insulin, HOMA-IR, PAL, or BMR.

In all subjects, after adjustment for age, PAL was significantly and negatively associated with waist circumference, fasting serum triglycerides, fasting serum insulin, and HOMA-IR (Table 2). These associations, except for the HOMA-IR association, remained significant even after further adjustment for BMI: PAL was significantly and negatively associated with waist circumference, fasting serum triglycerides, and fasting serum insulin. Neither systolic nor diastolic blood pressure was associated with PAL in the adjustment models.

Table 3 shows the standardized regression coefficients of PAL with the metabolic risk factors for the 38 male and 42 female subjects, respectively. In men, after adjustment for age, PAL was significantly and negatively associated with systolic blood pressure, FPG, fasting serum triglycerides, fasting serum insulin, and HOMA-IR. These associations, except for the fasting serum triglycerides association, remained significant after further adjustment for BMI: PAL was significantly and negatively associated with systolic blood pressure, FPG, fasting serum insulin, and HOMA-IR. In women, no significant associations were found between PAL and metabolic risk factors (Table 3).

## 4. Discussion

In the present study, we examined objectively the associations between daily physical activity and various metabolic risk factors. To our knowledge, this is the first study to investigate the associations between PAL measured by an accelerometer (and specifically a triaxial one) and metabolic risk factors in subjects with prediabetes (IFG and IGT) or untreated early T2D. We found in these populations that, after adjustment for age, PAL was significantly and negatively associated with waist circumference, fasting serum triglyceride and insulin levels, and HOMA-IR. These associations, except for the HOMA-IR association, remained significant even after further adjustment for BMI and thus suggest that higher PALs are favorably associated with abdominal obesity, hyperinsulinemia, and hypertriglyceridemia.

Our study also revealed sex differences in the associations between PAL and some of the metabolic risk factors. In an attempt to explain sex differences in the effects of PAL on some metabolic risk factors, we first looked at height and weight, which were both significantly greater in men than in women. After adjustment for age, height, and weight, PAL remained significantly and negatively correlated with systolic blood pressure, fasting serum insulin, and HOMA-IR in men, but not in women. This indicates that the sex differences in height and weight did not significantly influence the different effects of PAL on metabolic risk factors. These data agree with those after adjustment for BMI (Table 3). We looked next at BMR, which was significantly higher in men than in women. PAL determined by dividing TEE values by BMR values revealed no significant differences in PAL between men and women, indicating that PAL and BMR values cannot explain the sex differences in the effects of PAL on some metabolic risk factors. One reason why no significant associations were found between PAL and metabolic risk factors in women could be attributed to relatively small sample size. However, some physiological differences between men and women may explain our results. The average age of women was 58.9 ± 13.9 years, which suggests that most of female subjects were postmenopausal in the present study. Menopause is associated with decrease in muscle mass and strength, which is defined as sarcopenia [24], and the higher risk of falls [25]. Although no significant differences in PAL were observed between men and women, the amount of specific physical activity (i.e., locomotive activities such as walking and climbing stairs) might decrease in women. Previous epidemiological studies have demonstrated that walking is associated with a reduced risk of cardiovascular events [26, 27] and an improvement in 24 h glycemic control [28], suggesting that locomotive activities have the beneficial effects for metabolic risk factors. However, further research is needed to identify the potential mechanisms of sex differences in our study.

This study has several limitations. Its cross-sectional design does not allow for inferences of causality. Although we controlled for some confounding factors (age, sex, BMI, engagement in sports-like exercise or resistance training, and medication), other factors such as dietary intake change during study period and genetic variations were not taken into account. We aimed to measure light-intensity daily physical activity by the accelerometer but most of the subjects temporarily had moderate-intensity (≥3.0 METs) physical activity. However, mean PAL of study subjects was 1.64 (Table 1), indicating that they had sedentary or light activity lifestyle [23]. The heterogeneity of the study population of individuals with prediabetes (IFG and IGT) and T2D may also be a limitation. Actually, although serum triglycerides, serum insulin, and HOMA-IR were significantly higher in patients with T2D than in patients with prediabetes, no significant differences in physiological data such as age, BMI, or PAL were found between the two groups, and there were no significant associations between PAL and metabolic parameters within either group. To elucidate the associations between PAL and metabolic risk factors in patients with prediabetes or T2D, further larger scale studies are warranted. A limitation may exist with regard to the accelerometer used in this study. The triaxial accelerometer has been extensively validated for evaluating physical activity under free-living conditions [26, 29]; however, Leenders et al. showed that the predictive equations based on the relationship between acceleration and energy expenditure during locomotive movements leads to under- and overestimation of TEE [30]. It is possible therefore that energy expenditure and PAL measured using a triaxial accelerometer differ from the true values. In addition, PAL is not always equal to NEAT which we tried to evaluate by using the triaxial accelerometer, and further longitudinal studies will be needed to elucidate the associations between NEAT and metabolic risk factors.

## 5. Conclusion

In conclusion, among all subjects with prediabetes or untreated early T2D, higher objectively measured PAL was beneficially associated with waist circumference, serum triglycerides, and insulin resistance. In men, it was favorably associated with insulin resistance, FPG, and systolic blood pressure. Not only moderate-to-vigorous exercise but light-intensity daily physical activity is important in the management of patients with prediabetes and T2D.

## Figures and Tables

**Table 1:** Physical and biochemical characteristics of the subjects.

	All	Men	Women	*P* for sex difference
*n*	80	38	42	
Age (years)	57.6 ± 13.6	56.2 ± 13.4	58.9 ± 13.9	0.394
Height (cm)	160.6 ± 9.1	168.0 ± 6.0	153.9 ± 5.6	<0.001
Weight (kg)	68.0 ± 15.2	74.2 ± 14.7	62.4 ± 13.6	<0.001
BMI (kg/cm^2^)	26.2 ± 4.6	26.1 ± 3.8	26.3 ± 5.2	0.887
Waist circumference (cm)	92.0 ± 11.8	92.6 ± 10.8	91.4 ± 12.7	0.661
Systolic blood pressure (mmHg)	129.5 ± 17.2	127.8 ± 13.5	131.1 ± 20.0	0.401
Diastolic blood pressure (mmHg)	79.2 ± 12.5	78.5 ± 11.2	79.8 ± 13.6	0.642
Fasting plasma glucose (mg/dL)	121.1 ± 25.0	122.6 ± 26.6	119.7 ± 23.6	0.605
HbA1c (%)	6.7 ± 1.1	6.7 ± 1.2	6.6 ± 1.0	0.738
Total cholesterol (mg/dL)	213.6 ± 38.3	203.9 ± 33.6	222.3 ± 40.6	0.031
Triglycerides (mg/dL)	132.1 ± 92.5	124.1 ± 62.2	139.4 ± 113.5	0.463
HDL cholesterol (mg/dL)	53.5 ± 15.7	50.6 ± 17.2	56.1 ± 13.9	0.116
LDL cholesterol (mg/dL)	127.3 ± 44.2	128.5 ± 28.1	126.3 ± 54.3	0.204
Serum insulin (*μ*U/mL)	9.7 ± 6.6	9.8 ± 7.5	9.6 ± 5.7	0.844
HOMA-IR	3.0 ± 2.4	3.2 ± 3.0	2.9 ± 1.8	0.563
Physical activity level	1.64 ± 0.17	1.63 ± 0.16	1.64 ± 0.17	0.485
Basal metabolic rate (kcal/day)	1318.9 ± 272.4	1499.9 ± 225.5	1115.3 ± 198.4	<0.001

Data are expressed as means ± SD. HDL: high-density lipoprotein; LDL: low-density lipoprotein; HOMA-IR: homeostasis model assessment-insulin resistance.

**Table 2:** Standardized regression coefficients of physical activity levels with metabolic risk factors in 80 adults with prediabetes or type 2 diabetes.

All subjects	Adjusted for age		Adjusted for age and BMI	
	Standardized regression coefficient	*P* value	Standardized regression coefficient	*P* value
	(95% CI)		(95% CI)	
Waist circumference (cm)	−0.238 (−0.448 to −0.028)	0.027	−0.124 (−0.226 to −0.022)	0.018
Systolic blood pressure (mmHg)	−0.063 (−0.290 to 0.204)	0.582	−0.021 (−0.243 to 0.201)	0.851
Diastolic blood pressure (mmHg)	−0.133 (−0.352 to 0.086)	0.230	−0.093 (−0.304 to 0.118)	0.383
Fasting plasma glucose (mg/dL)	−0.063 (−0.291 to 0.165)	0.584	−0.044 (−0.273 to 0.185)	0.703
Triglycerides (mg/dL)	−0.253 (−0.473 to −0.033)	0.024	−0.239 (−0.461 to −0.017)	0.035
Serum insulin (*μ*IU/mL)	−0.279 (−0.486 to −0.072)	0.009	−0.224 (−0.414 to −0.034)	0.022
HOMA-IR	−0.240 (−0.451 to −0.029)	0.026	−0.193 (−0.392 to 0.006)	0.058

Data are expressed as the means ± SD. BMI: body mass index; CI: confidence interval; HOMA-IR: homeostasis model assessment-insulin resistance.

**Table 3:** Standardized regression coefficients of physical activity levels with metabolic risk factors in men and women with prediabetes or type 2 diabetes.

	Adjusted for age		Adjusted for age and BMI	
	Standardized regression coefficient	*P* value	Standardized regression coefficient	*P* value
	(95% CI)		(95% CI)	
Men (*n* = 33)				
Waist circumference (cm)	−0.290 (−0.602 to 0.022)	0.067	−0.098 (−0.216 to 0.02)	0.113
Systolic blood pressure (mmHg)	−0.381 (−0.722 to −0.04)	0.026	−0.351 (−0.693 to −0.009)	0.044
Diastolic blood pressure (mmHg)	−0.309 (−0.646 to 0.028)	0.071	−0.269 (−0.611 to 0.073)	0.119
Fasting plasma glucose (mg/dL)	−0.422 (−0.739 to −0.15)	0.011	−0.369 (−0.689 to −0.049)	0.025
Triglycerides (mg/dL)	−0.348 (−0.680 to −0.105)	0.040	−0.302 (−0.641 to 0.037)	0.079
Serum insulin (*μ*IU/mL)	−0.279 (−0.486 to −0.016)	0.004	−0.362 (−0.640 to −0.084)	0.012
HOMA-IR	−0.460 (−0.761 to −0.159)	0.004	−0.371 (−0.652 to −0.09)	0.011
Women (*n* = 42)				
Waist circumference (cm)	−0.241 (−0.571 to 0.089)	0.147	−0.161 (−0.327 to 0.005)	0.057
Systolic blood pressure (mmHg)	−0.037 (−0.377 to 0.303)	0.827	−0.001 (−0.255 to 0.253)	0.994
Diastolic blood pressure (mmHg)	−0.067 (−0.390 to 0.256)	0.677	−0.034 (−0.341 to 0.273)	0.824
Fasting plasma glucose (mg/dL)	0.104 (−0.243 to 0.035)	0.548	0.108 (−0.244 to 0.46)	0.538
Triglycerides (mg/dL)	−0.243 (−0.578 to 0.092)	0.151	−0.237 (−0.578 to 0.104)	0.167
Serum insulin (*μ*IU/mL)	−0.098 (−0.415 to 0.219)	0.535	−0.059 (−0.348 to 0.23)	0.682
HOMA-IR	−0.038 (−0.359 to 0.283)	0.812	−0.006 (−0.333 to 0.321)	0.971

Data are expressed as the means ± SD. BMI: body mass index; CI: confidence interval; HOMA-IR: homeostasis model assessment-insulin resistance.
